# Matrix Metalloproteinase-3 in Odontoblastic Cells Derived from Ips Cells: Unique Proliferation Response as Odontoblastic Cells Derived from ES Cells

This article has been retracted.

**DOI:** 10.1371/journal.pone.0083563

**Published:** 2013-12-16

**Authors:** Taiki Hiyama, Nobuaki Ozeki, Makio Mogi, Hideyuki Yamaguchi, Rie Kawai, Kazuhiko Nakata, Ayami Kondo, Hiroshi Nakamura

**Affiliations:** 1 Department of Endodontics, School of Dentistry, Aichi Gakuin University, Nagoya, Aichi, Japan; 2 Department of Medicinal Biochemistry, School of Pharmacy, Aichi Gakuin University, Nagoya, Aichi, Japan; The University of Hong Kong, Hong Kong

## Abstract

We previously reported that matrix metalloproteinase (MMP)-3 accelerates wound healing following dental pulp injury. In addition, we reported that a proinflammatory cytokine mixture (tumor necrosis factor-α, interleukin (IL)-1β and interferon-γ) induced MMP-3 activity in odontoblast-like cells derived from mouse embryonic stem (ES) cells, suggesting that MMP-3 plays a potential unique physiological role in wound healing and regeneration of dental pulp in odontoblast-like cells. In this study, we tested the hypothesis that upregulation of MMP-3 activity by IL-1β promotes proliferation and apoptosis of purified odontoblast-like cells derived from induced pluripotent stem (iPS) and ES cells. Each odontoblast-like cell was isolated and incubated with different concentrations of IL-1β. MMP-3 mRNA and protein expression were assessed using RT-PCR and western blotting, respectively. MMP-3 activity was measured using immunoprecipitation and a fluorescence substrate. Cell proliferation and apoptosis were determined using ELISA for BrdU and DNA fragmentation, respectively. siRNA was used to reduce MMP-3 transcripts in these cells. Treatment with IL-1β increased *MMP-3* mRNA and protein levels, and MMP-3 activity in odontoblast-like cells. Cell proliferation was found to markedly increase with no changes in apoptosis. Endogenous tissue inhibitor of metalloproteinase (TIMP)-1 and TIMP-2 were constitutively expressed during all experiments. The exocytosis inhibitor, Exo1, potently suppressed the appearance of MMP-3 in the conditioned medium. Treatment with siRNA against MMP-3 suppressed an IL-1β-induced increase in MMP-3 expression and activity, and also suppressed cell proliferation, but unexpectedly increased apoptosis in these cells (*P*<0.05). Exogenous MMP-3 was found to induce cell proliferation in odontoblast-like cells derived from iPS cells and ES cells. This siRNA-mediated increase in apoptosis could be reversed with exogenous MMP-3 stimulation (*P*<0.05). Taken together, IL-1β induced MMP-3-regulated cell proliferation and suppressed apoptosis in odontoblast-like cells derived from iPS and ES cells.

## Introduction

Since matrix metalloproteinases (MMPs), a family of calcium and zinc-dependent extracellular matrix (ECM) degrading enzymes, are expressed in physiological and pathophysiological processes, and process virtually any component of the ECM, it has been suggested that MMPs may be important in inflammatory conditions such as rheumatoid arthritis and periodontitis where they participate in inflammation [1]–[4]. There are no basal levels of MMP-3 mRNA and protein in cells, and MMP-3 synthesis is tightly controlled *in vivo*. Significantly elevated levels of MMP-1, MMP-2 and MMP-3 have been detected in acute and chronic rheumatoid arthritis, inflamed pulps and in periapical lesions when compared with healthy tissues [1], [5]–[7]. While it is intuitive that dental pulp destruction may be a function of MMPs, our previous study reported that MMP-3 actually accelerates wound healing following dental pulp injury. This observation indicates that MMP-3 may be involved in both ECM degradation and the subsequent morphogenesis, wound repair [8], [9] and angiogenesis in the inflamed tissue [10]–[12].

The regulation of metalloproteinases is very complex. Regulation occurs at different levels and on a broader scale, three levels of endogenous control exist: transcriptional regulation, zymogen activation and regulation on the level of enzymatic activity by different endogenous regulators. A wide variety of cytokines, growth factors and oncogene products stimulate MMP expression [13], [14]. Tumor necrosis factor (TNF)-α and interleukin (IL)-1 are regularly involved in metalloproteinase gene induction [15]–[18]. Although we previously reported that a proinflammatory cytokine mixture (IL-1β, TNF-α, and IFN-γ) could induce MMP-3 activity in odontoblast-like cells derived from mouse embryonic stem (ES) cells [19], the identification of the principal cytokine responsible for this MMP-3 stimulus remains unresolved. As a trophic factor, the multifunctional cytokine IL-1 plays an important role in the proliferation of cells at the site of tissue injury [1], [20]; although the signals that control cells from proliferation during wound healing are unclear. In general, a relatively low level of IL-1 can induce cell proliferation; however, high levels of the cytokine cause apoptotic cell death [21]–[23]. Given that IL-1β has been detected in inflamed dental pulps and was associated with periapical disease [24], this cytokine was believed to be essential in the pathogenesis of pulpitis. In particular, treatment with IL-1β resulted in the potent induction of *MMP-3* expression in dental pulp, which contains large numbers of odontoblasts [7]. Taken together, these studies suggest that MMP-3 induced by the proinflammatory cytokine IL-1β contributes to the pathophysiology of inflamed dental pulp. In particular, the dental pulp tissue consists predominantly of odontoblasts, with small populations of fibroblasts, blood vessels and neurons [25], therefore, odontoblasts may represent a new target for therapeutic strategies. Due to the challenges associated with obtaining sufficient amounts of purified odontoblast cells, no study has focused on odontoblast cells following the induction of inflammation. The heterogeneous nature of cells in the dental pulp obfuscates direct investigation of MMP-3 effects in whole dental pulp. Moreover, while the development of our basic knowledge with regard to stem cell differentiation is highly valuable, the use of human ES cells is ethically controversial and treatments employing these cells are unlikely to be realized in the near future. Consequently, we undertook our experiments using purified odontoblast-like cells derived from induced pluripotent stem (iPS) cells [26] and ES cells [27], which are excellent models in which to examine the mechanism of wound healing *in vitro*.

We have addressed several points described above using odontoblast-like cells derived from mouse iPS cells and ES cells.Here, we focus on the relationship between IL-1β-induced MMP-3 accumulation and the responses of odontoblast-like cells derived from iPS cells and ES cells *in vitro*. We used siRNA directed against *MMP-3* transcripts to examine whether IL-1β-induced changes in cell proliferation and apoptosis of odontoblast-like cells derived from iPS cells is associated with an increase in the expression and activity of MMP-3.

## Materials and Methods

### Materials

Mouse recombinant IL-1β was obtained from PeproTech (Rocky Hill, NJ, USA).

Recombinant human MMP-3 was obtained from Chemicon (Temecula, CA, USA). Exocytotic inhibitor (Exo) 1 and 2-(4-Fluorobenzoylamino) methylbenzoate, an inhibitor of protein trafficking emanating from the ER, which acts by inducing the rapid collapse of the Golgi, were obtained from Sigma-Aldrich (St. Louis, MO, USA).

### Cell cultures

The mouse iPS cell line iPS-MEF-Ng-20D-17 [28] was a gift from Prof. Yamanaka (Kyoto, Japan) and was maintained as described previously [28], [29]. An E14Tg2a ES cell [30] was a kind gift from Dr. Randall H. Kramer (UCSF, San Francisco, CA, USA) and maintained as described previously [31]. Moreover, B6G-2 ES cells were from the Riken cell bank (Ibaraki, Japan) and were maintained as described previously [32]. B6G-2 cells require feeders, whereas E14Tg2a cells do not require feeders, thus both cells were used for comparison. Rat odontoblast-like cells (KN-3 [33]; kindly provided by Dr. Chiaki Kitamura, Kyushu Dental College, Kitakyushu, Japan) were maintained as described previously [33] and used as an authentic control. Purified odontoblast-like cells derived from ES cells [27] were prepared as reported previously [27]. Purified odontoblast-like cells derived from iPS cells were also prepared as reported [26]. The monoclonal anti-α2 integrin antibody is known to potently suppress the expression of odontoblastic markers in these cultured systems. Thus, we could confirm that the expression of α2 integrin in ES cells triggered their differentiation into odontoblast-like cells [27]. The proportion of α2 integrin-positive cells in the total differentiated odontoblast-like cell population is a measure of the purity of the B6G-2- and E14Tg2a-derived odontoblast-like cells, and was estimated by FACS analysis to be 98.63±0.74% (iPS-derived odontoblast-like cells; *n* = 3), 98.53±0.88% (B6G-2-derived odontoblast-like cells; *n* = 3), or 98.79±0.43% (E14Tg2a-derived odontoblast-like cells; *n* = 3). The resultant differentiated cells were shown to have odontoblast-like physiological characteristics (e.g., calcification activity and alkaline phosphatase activation) up to day 21 of the culture.

### Determination of apoptotic cell death by ELISA

Cellular DNA fragmentation was assessed by detection of BrdU-labeled DNA fragments in the cytoplasm of cell lysates using solid-phase-immobilized anti-DNA monoclonal antibodies and anti-BrdU monoclonal antibodies labeled with peroxidase (Cellular DNA fragmentation ELISA; Roche Applied Science, Mannheim, Germany), according to the manufacturer's instructions and previously published studies [22], [34], [35].

### Cell proliferation assay

Cell proliferation was evaluated using the BrdU-cell proliferation ELISA (Roche Applied Science, Mannheim, Germany) as described previously [22], [34], [35]. The cells were seeded into 96-well tissue culture plates at a density of 1×10^5^ cells/cm^2^.

### Semi-quantitative reverse transcription polymerase chain reaction (RT-PCR) analysis

The cells were seeded into 6-well tissue culture plates at a density of 1×10^5^ cells/cm^2^. The cells were cultured for 2 h with or without IL-1β, and total RNA was isolated from the cultured cells using an RNeasy Mini Kit (Qiagen, Inc., Valencia, CA, USA). The amount of RNA was equalized using a glyceraldehyde 3-phosphate dehydrogenase (GAPDH) competitive PCR kit (Takara Shuzo Co., Shiga, Japan). The mRNA was converted to complementary DNA (cDNA) with the GeneAmp RNA PCR kit (Perkin Elmer, Branchburg, NJ, USA). The primer sequences and sizes, and accession numbers of the amplicons are as follows: rat MMP-3 (sense 5′-cctgagaccttaccaatgtgtagc-3′, antisense 5′-caacatggatgctgcatatgaagtt-3′; 189-bp amplicon, NM_133523), mouse MMP-3 (sense 5′-aggatttcccaggaagatagctgag-3′, antisense 5′-aattccaacagcgaagatccact-3′; 114-bp amplicon, NM_010809), mouse TIMP-1 (sense 5′-cagcaaagagctttctcaaagacct-3′, antisense 5′-tagataaacagggaaacactgtgca-3′; 70-bp amplicon, NM_011593), mouse TIMP-2 (sense 5′-ggacctgacaaagacttcgagttta-3′, antisense 5′-ccatctccttctgcctttcctg-3′; 119-bp amplicon, NM_011594), rat GAPDH (sense 5′-gctctctgctcctccctgttc-3′, antisense 5′-cgtccgatacggccaaatcc-3′; 113 bp amplicon, NM_017008) and mouse GAPDH (sense 5′-aatggtgaaggtcggtgtgaac-3′, antisense 5′-cgtgagtggagtcggaac-3′; 155-bp amplicon, NM_008084). The primer mixture, a total volume of 25 µl, contained 50 µM deoxynucleoside triphosphates, 0.5 units of Tag DNA polymerase, 1.5 mM MgCl_2_ and 1 µM of forward and reverse primers in a 10× PCR reaction buffer (200 mM Tris-HCl, 500 mM KCl, pH 8.3). The PCR reaction within the exponential phase of the amplification curve was performed for 25 cycles for MMP-3, TIMP-1, TIMP-2 and GAPDH under the following conditions: initial denaturation at 94°C for 2 min, denaturation at 94°C for 30 s, annealing at 64°C for rat MMP-3, at 67°C for mouse MMP-3, at 66°C for mouse TIMP-1, at 66°C for mouse TIMP-2, at 61°C for rat GAPDH and at 65°C for mouse GAPDH for 30 s, and an extension period at 72°C for 1 min. The PCR products were loaded in a 1.5% agarose gel, visualized with ethidium bromide and photographed. The intensities of the PCR products were quantified using a scanner and digital image analysis software (Multi Gauge-Ver3.X, Fujifilm, Tokyo, Japan).

### Western blot analysis

MMP-3 protein levels in the cell lysate were determined by western blot analysis. Cells were cultured for 6 h with or without IL-1β, lysed and the protein lysate separated on SDS-polyacrylamide gels (12%) in preparation for western blot analysis using anti-MMP-3, anti-TIMP-1, anti-TIMP-2 and b-tubulin polyclonal antibodies (sc-6839, sc-5538, sc-6835 and sc-9935, respectively; Santa Cruz Biotechnology, Inc., Santa Cruz, CA, USA). The anti-MMP-3 antibody showed no significant cross-reactivity with other MMPs (data not shown). Visualization and quantification of blotted protein bands were performed with the Multi Gauge-Ver3.X software (Fujifilm).

### Measurement of MMP-3 activity

The protocol for measuring MMP-3 activity was described previously [36] and has been incorporated into a commercially available MMP-3 activity assay kit (SensoLyte™ 520 MMP-3 assay kit; AnaSpec, San Jose, CA, USA). Prior to detection, MMP-3 was immunoprecipitated from the culture medium using a goat anti-MMP-3 antibody (sc-6839, Santa Cruz Biotechnology, Inc.) and protein A/G–agarose for 6 h at 4°C. After centrifugation, the agarose pellets were suspended in a MMP-3 assay buffer (containing the MMP-3 substrate as 5-Carboxyfluorescein (FAM)/Arg-Pro-Lys-Pro-Val-Glu-Nva-Trp-Arg-Lys-QXL™ 520-NH2 fluorescence resonance energy transfer (FRET) [37], [38] peptide) supplied in the assay kit, and the activity of MMP-3 was determined according to the manufacturer's instructions.

### Silencing of the MMP-3 gene by siRNA transfection

The anti-MMP-3 siRNAs for gene silencing were acquired commercially (sc-37265 and sc-61874, Santa Cruz Biotechnology, Inc.) and transfected into cultured cells using a siRNA reagent system (Santa Cruz Biotechnology, Inc.) according to the manufacturer's protocol. An anti-GAPDH siRNA and a siRNA with no known homogeny for any vertebrate sequence (Thermo Scientific, Lafayette, CO, USA) were used as positive and negative controls, respectively.

### Statistical analysis

Data are presented in bar graphs are the means ± standard deviations (SD) of 4–6 independent experiments. Statistical significance was assessed using the Mann-Whitney U-test. *P*<0.05 was considered as statistically significant.

## Results

### IL-1b induces the expression of MMP-3 mRNA and protein, and MMP-3 activity in odontoblast-like cells

The odontoblast-like cells derived from iPS cells, ES cells and KN-3 were cultured in the presence of three concentrations of IL-1β (0, 0.25, 2.5 and 25 ng/mL) and MMP-3 induction was assessed using RT-PCR and western blot analysis. We found that 0.25 and 2.5 ng/mL IL-1β induced *MMP-3* mRNA and protein expression, whereas 25 ng/mL IL-1β did not affect MMP-3 levels (Figure 1A and 1B).

**Figure 1:** The increased expression of *MMP-3* mRNA and MMP-3 protein in odontoblast-like cells. (A) Increased expression of *MMP-3* and *GAPDH* (a housekeeping gene) transcripts measured using RT-PCR. (B) Western blot analysis of the levels of MMP-3 and β-tubulin. The β-tubulin protein served as the internal control to confirm that equal amounts of the total protein extract had been loaded into each well of the gel. Each experiment was repeated three times and the results shown are representative of these three independent experiments.

MMP-3 activity is precisely regulated at the level of transcription by the activation of their precursor zymogens, and by the action of endogenous inhibitors, namely TIMPs [39]. Although it in known that TIMP-2 is inducible by cytokines [39], we confirmed that both TIMP-1 and TIMP-2 mRNA and protein levels were constitutively expressed in all experimental conditions (Figure 2). To normalize the increase in MMP activity, it is necessary to describe the activity in the context of TIMP protein expression. As shown in Figure 2, TIMP-1 and TIMP-2 were present continuously at stable levels under all experimental conditions. To assess the intracellular MMP-3 peptidase activity induced by IL-1β treatment, we assayed MMP-3 activity in immunoprecipitates prepared from cell culture medium following cell treatment with various concentrations of extracellular IL-1β (0, 0.25, 2.5 and 25 ng/mL). We observed significant increases in MMP-3 activity in the culture medium from cells treated with 0.25 and 2.5 ng/mL of cytokine, but not in that from cells treated with 25 ng/mL of IL-1β (*P*<0.01; Figure 3), as compared with control cultures.

**Figure 2:** IL-1β induces the expression of TIMP mRNA and TIMP in odontoblast-like cells. (A) Expression of *TIMP-1, TIMP-2* and *GAPDH* (housekeeping gene) transcripts measured using RT-PCR. (B) Western blot analysis of TIMP-1 and TIMP-2 protein expression in each cell line. Data are representative of at least three independent experiments.

**Figure 3:** Effect of exogenous IL-1β on MMP-3 activity in odontoblast-like cells. Effect of exogenous IL-1β on MMP-3 activity in odontoblast-like cells derived from iPS cells, ES cells and KN-3, as evaluated by the immunoprecipitation-MMP-3 assay. The cells were incubated in serum-free medium in the absence or presence of IL-1βfor the times indicated (6 h  =  white bars, or 12 h  =  black bars). Data are presented as the mean ± SD of six independent experiments; (vs. control, *P<0.05).

The level of mRNA (Figure 1A) is somewhat irrelevant because it does not give any information about how the MMP-3 is released once it is made, i.e., it could be released exocytically or by cell death. When we performed a simple experiment in the presence and absence of an exocytosis inhibitor, such as Exo1, to demonstrate that inhibiting exocytosis precludes the appearance of MMP-3 in the conditioned medium, we demonstrate that Exo1 (3 µM) could attenuate the appearance of MMP-3 in the conditioned medium (Figure 4). Therefore, we confirmed that IL-1β-induced MMP-3 is released exocytically from these cells.

**Figure 4:** Effects of exocytosis inhibitor Exo1 treatment with IL-1β on MMP-3 activity in odontoblast-like cells. The cells were incubated in serum-free medium in the absence or presence of Exo1 (0, 1, or 3 µM) and IL-1βfor the times indicated (6 h  =  grey bars, or 12 h  =  black bars). Data are presented as the mean ± SD of four independent experiments;. (**P<0.01 *vs*. control; ^#^ *P*<0.05 *vs*. Exo1 (1 µM); ^†^ *P*<0.01, as indicated by the bracket).

### Effect of exogenous IL-1β on DNA fragmentation and cell proliferation in odontoblast-like cells

We next sought to assess the effect of IL-1β on MMP-3-mediated apoptosis and cell proliferation. At 25 ng/mL, IL-1β was found to induce a significant (>400%) increase in apoptosis (*P*<0.01; Figure 5A) and a decrease in proliferation (Figure 5B). The lower concentrations of exogenous IL-1β (0.25 and 2.5 ng/mL) were found to increase cell proliferation of odontoblast-like cells derived from iPS cells, ES cells and KN-3 (*P*<0.05; Figure 5B) and apoptotic cell death was not detected (Figure 5A). Since apoptosis and proliferation rates appear to be inversely correlated, the increase in apoptosis induced by the IL-1β at a concentration of 25 ng/mL may cause a marked decrease in proliferation observed in these odontoblast-like cells under these conditions.

**Figure 5:** Effect of exogenous IL-1β on DNA fragmentation and cell proliferation in odontoblast-like cells. (A) Effect of exogenous IL-1β on DNA fragmentation in odontoblast-like cells derived from iPS cells, ES cells, and KN-3, as evaluated by the detection of BrdU-labeled DNA fragments. Data are presented as the mean ± SD of six independent experiments; (vs. control, *P<0.05, **P<0.01). (B) Effect of exogenous IL-1β on cell proliferation, as evaluated using the BrdU-cell proliferation ELISA. The cells were incubated in the absence or presence of IL-1β (0, 0.25, 2.5, and 25 ng/mL) for 24 h. Data are presented as the mean ± SD of at four independent experiments; (vs. control, *P<0.05, **P<0.01).

### Effect of MMP-3 siRNA on IL-1b-induced MMP-3 expression in odontoblast-like cells

We next employed siRNA directed against MMP-3 to determine if the effects observed with IL-1β stimulation were mediated by MMP-3 in each cell type. Cells were transfected with MMP-3 siRNA or a control siRNA and then stimulated with IL-1β as described above. *MMP-3* was expressed in cells transfected with control siRNA but not in cells transfected with the MMP-3 siRNA (Figure 6A). We observed no change in the expression of the internal control (*GAPDH*) after transfection, and the negative control siRNA confirmed that the effect on the cells was specific to MMP-3. Moreover, western blot analysis confirmed the efficient silencing of the MMP-3 gene at the protein level in the presence of IL-1β stimulation (Figure 6B). Transfection with siRNA had no effect on the level of expression of β-tubulin, which was used as a control to ensure equal loading.

**Figure 6:** The effect of transfection of odontoblast-like cells with siRNA on the levels of MMP-3. (A) RT-PCR analysis of the *MMP-3* gene expression in cells 24 h after transfection with siRNA. (B) Western blot analysis of the increased expression of MMP-3 in cells 24 h after transfection with siRNA. Each experiment was repeated three times and the results shown are representative of these three independent experiments.

### Effect of MMP-3 siRNA on IL-1β-induced MMP-3 activity in odontoblast-like cells

Next, we demonstrated that transfection of MMP-3 siRNA also efficiently down-regulated MMP-3 activity (*P*<0.01; Figure 7). The control siRNA had no effect on the changes in *MMP-3* mRNA, MMP-3 protein levels, or MMP-3 activity induced by IL-1β (0.25 and 2.5 ng/mL; Figure 7).

**Figure 7:** The effect of transfection of odontoblast-like cells with siRNA on the levels of MMP-3 activity. Effects of the combination of IL-1β treatment (0, 0.25, 2.5 and 25 ng/mL) on MMP-3 activity released from cultured cells 24 h after transfection with siRNA. The cells were incubated in serum-free medium in the absence or presence of exogenous IL-1β at the concentrations indicated for either 6 h (white bars) or 12 h (black bars). Data are presented as the mean ± SD of four independent experiments. *, ^#^ and ^†^ denote significant differences; (*P<0.05 *vs*. control; ^#^ *P*<0.05 *vs*. control siRNA; ^†^ *P*<0.01, as indicated by the bracket).

### Effect of MMP-3 siRNA on DNA fragmentation and cell proliferation in odontoblast-like cells

Under the same culture conditions described above, we next tested the effect of MMP-3 siRNA on IL-1β–induced changes in apoptosis and cell proliferation. Silencing the MMP-3 gene considerably increased the number of apoptotic cells compared with the non-transfected control group following treatment with the IL-1β. The degree of apoptotic cell death in MMP-3 siRNA-transfected cells treated with the cytokine was 3-fold higher than in the non-transfected control group (*P*<0.01; Figure 8). There was no such increase in apoptosis in cells treated with the control siRNA. The control siRNA did not attenuate the cell proliferation induced by IL-1β (0.25 and 2.5 ng/mL) (Figure 9). The number of cells with proliferative potential was 60% less in MMP-3 siRNA-transfected cells than in non-transfected cells (*P*<0.05; Figure 9).

**Figure 8:** Effect of MMP-3 siRNA on DNA fragmentation in odontoblast-like cells. DNA fragmentation of the cells 24-3 evaluated by the detection of BrdU-labeled DNA fragments; (**P<0.01 *vs*. control; ^##^ *P*<0.01 *vs*. control siRNA; ^†^ *P*<0.01, as indicated by the bracket.) Data are presented as the mean ± SD of six independent experiments.

**Figure 9:** Effect of MMP-3 siRNA on cell proliferation in odontoblast-like cells. Cell proliferation of odontoblast-like cells derived from iPS cells, ES cells and KN-3 24 h after transfection with siRNA designed to target MMP-3 evaluated using BrdU-cell proliferation ELISA; (**P<0.01 *vs*. control; ^##^ *P*<0.01 *vs*. control siRNA; ^†^ *P*<0.01 as indicated by the bracket). Data are presented as the mean ± SD of six independent experiments.

### Effect of exogenous MMP-3 on cell proliferation in odontoblast-like cells

We tested whether exogenous MMP-3 could enhance proliferation in odontoblast-like cells derived from iPS cells. Interestingly, the addition of MMP-3 (10, 30, or 50 ng/mL) increased cell proliferation (*P*<0.05; Figure 10) in a dose-dependent manner, but caused a dramatic decrease in cell proliferation at the highest concentration tested (100 ng/mL) (Figure 10). Exogenous MMP-3 also induced cell proliferation in odontoblast-like cells from ES cells and rat KN-3.

**Figure 10:** Effect of exogenous MMP-3 on cell proliferation in odontoblast-like cells. Effects of exogenous MMP-3 on odontoblast-like cells proliferation derived from iPS cells, ES cells and KN-3. Cells were incubated in serum-free medium in the absence or presence of various concentrations of MMP-3 (0, 10, 30, 50 and 100 ng/mL) for 24 h prior to cell proliferation evaluation using the BrdU-cell proliferation ELISA. Data are the mean ± SD of six independent experiments; (vs. control, *P<0.05, **P<0.01).

### Effect of exogenous MMP-3 on IL-1 β induced DNA fragmentation in odontoblast-like cells

Finally, we next tested whether exogenous MMP-3 could rescue the apoptotic effects seen with MMP-3 siRNA. Our results confirmed that exogenous MMP-3 (5, 10, 20 and 30 ng/ml) could rescue the cells from undergoing IL-1β-induced apoptosis (0.25 ng/ml) in the presence of MMP-3 siRNA (*P*<0.01; Figure 11).

**Figure 11:** Effects of exogenous MMP-3 on odontoblast-like cells apoptosis induced by IL-1βandMMP-3 siRNA treatment. Cells were incubated in serum-free medium in the absence or presence of MMP-3 (5, 10, 20 and 30 ng/mL), and MMP-3 siRNA combined with IL-1β (0 and 0.25 ng/mL) for 24 h, and then DNA fragmentation (i.e., apoptosis index) was evaluated by the BrdU-labeled DNA fragmentation ELISA. Data are the mean ± SD of six independent experiments; (vs. as control with the IL-1βaddition (0.25 ng/mL), **P<0.01, ^†^ *P*<0.05 as indicated by the bracket).

## Discussion

Currently, the effects of suppression of MMP-3 activity on the apoptosis of odontoblast-like cells derived from iPS cells has not been reported previously, because purified odontoblast-like cells were not available. In our previous report, a cytokine mixture induced MMP-3 regulated cell proliferation and suppressed apoptosis in mouse ES cells derived odontoblast-like cells [19]. IL-1β also induces MMP-3-regulated cell proliferation and suppresses apoptosis in rat dental pulp cells [40]. However, as dental pulp cells consist of fibroblasts, odontoblast cells, vessels and neuronal cells in the tissue [25], it was unclear which cells were mainly regulated by IL-1β-induced MMP-3. In the current study, IL-1β was found to activate MMP-3 in odontoblast-like cell, and this observation represents a novel physiological function of MMP-3.

Our data highlights four main points. First, this is the first report that involved the use of siRNA that targets *MMP-3* to elucidate the mechanism on IL-1β-induced proliferation of odontoblast-like cells derived from iPS and ES cells. Given the challenges of obtaining sufficient amounts of purified odontoblast-like cells, this is the first study to investigate odontoblast-like cells after induction with a proinflammatory cytokine. As shown in the method described above, the purity of these cells was ∼98% and the cells display the physiological functions of odontoblast-like cells. It is likely that the characterization of the cells derived from iPS cells is different from the one derived from ES cells. Since odontoblast-like cells derived from iPS cell showed similar responses as those observed for odontoblast-like cells derived from ES cells [19], we demonstrated a good correlation and the availability of two-cell lines to produce odontoblast-like cells. Secondly, since we confirmed that a relatively low amount of exogenous MMP-3 (30 and 50 ng/mL) increases cell proliferation (Figure 10) and rescues cells from undergoing apoptosis (MMP-3: 5–30 ng/mL; Figure 11), it is possible that minor accumulation of MMP-3 stimulates the regulation of cell proliferation within a microenvironmental site (e.g., at sites of inflammation). Thirdly, since we demonstrated that a cytokine mixture induced MMP-3 also regulated cell proliferation of odontoblast-like cells from ES cells [19], the effects of the cytokine mixture on the odontoblast-like cells may be primarily due to the presence of IL-1β. Finally, while relatively high amounts of IL-1β caused apoptotic cell death with no induction of MMP-3, low amounts of IL-1β could produce MMP-3 in the cells tested. Although IL-1-induce MMPs are involved in the breakdown of ECM in disease processes, such as arthritis and tumor metastasis [11], [41]–[43], there is no MMP-3 mRNA and MMP-3 under normal physiological conditions because of the absence of the required cytokines to stimulate production of this protein, as shown in Figure 1. Taken together, the physiological function of IL-1β-induced MMP-3 might play a role in anti-apoptotic activity, but not a destructive role in cells during the early phase of inflammation.

It remains to be established how IL-1β-induced MMP-3 activity regulates the anti-apoptotic effect of odontoblast-like cells. We hypothesize that, with so much apoptosis occurring as shown in Figure 5 and 8, there may also be a limited amount of uncontrolled cell death that leads to the release of MMP-3 into the conditioned medium. To test this concept we measured MMP-3 levels in the presence and absence of an exocytosis inhibitor, Exo1, to demonstrate that shutting down exocytosis suppressed the appearance of MMP-3 in the conditioned medium (Figure 4). Taken together, we believe that the presence of MMP-3 in the culture corresponds to exocytosis of the enzyme, and not to passive output as a consequence of cell death.

It is unclear how cytokine-induced MMP-3 regulates odontoblast-like cells proliferation and what molecular pathways upregulate MMP-3 following exposure to IL-1β. Recent reports demonstrated that IL-1β-induced MMP-3 is associated with the secreted glycoprotein Wnt signal pathway [44]. Blockage of JNK signaling impairs the Wnt-5A-induced up-regulation of MMP-3. Thus, Wnt-5A may be associated with cartilage destruction by promoting the expression of MMP-3 [45]. MMP-3 also induces hyperplastic mammary epithelial growth and regulates Wnt signaling by antagonizing Wnt-5B function [46]. The nature of the pathway by which MMP-3 induces cell proliferation, however, remains to be elucidated.

Although MMP activity is but one factor that regulates the destruction of tissue, our previous study demonstrated that MMP-3 accelerates wound healing following dental pulp injury [8], [9]. We also confirmed that the exogenous MMP-3 could induce cell proliferation in odontoblast-like cells (Figure 10). Taken together with our previous report, the current evidence suggests that lower concentrations of IL-1β can induce MMP-3-drived increases in odontoblast-like cell proliferation, whereas higher concentrations inhibit cell proliferation and promote apoptosis.
